The article "Visual Sensor Image Analysis and Massage Techniques to Prevent and Treat Common Injuries of Sports Dance Practitioners" was retracted in 2023. Reasons: signs of a paper mill; suspected computer-generated content; unreliable results or conclusions; concerns about the data.

# Visual Sensor Image Analysis and Massage Techniques to Prevent and Treat Common Injuries of Sports Dance Practitioners

**DOI:** 10.1155/2022/5665972

**Published:** 2022-02-07

**Authors:** Chengxuan Yu, Ru Li

**Affiliations:** Zhengzhou Shengda University of Economics, Business & Management, Zhengzhou 450000, Henan, China

## Abstract

In recent years, the performance of sports dance in China has become better and better. Naturally, the technical requirements for this dance are getting higher and higher, and the number and intensity of training have also increased, which has led to increasing injuries in sports dance. This article is based on visual sensor images to analyze and study the common injuries and prevention of sports dance practitioners. It is aimed at providing a certain reference basis for athletes' injuries, so that dance practitioners and coaches can better master sports dance training and teaching. Injury-related rules and prevention reduce the injury rate. This article puts forward the related technology of a visual sensor image and applies its technology to the prevention and research of common injuries in sports dance. At the same time, it analyzes the causes of sports dance practitioners' injuries and seeks economical and affordable massage techniques for prevention, and the method of treatment provides protection for dance practitioners. The experimental results in this article show that the Tuina group cured 15 subjects, 41 subjects were markedly effective, 13 subjects were improved, and 6 subjects were unhealed. The total effective rate was 92%.

## 1. Introduction

### 1.1. Background

Sports dance is a national standard that people often say. This combines dance, art, and competitive sports. As an art form, it perfectly reflects the unique artistic value of decoration and dance as well as excellent body function. Whether it is a dance art project or a sports project, there is almost no sports dance that can perfectly integrate entertainment, fitness, performance, and competition, but sports dance has done it. With its unique dancing posture and passionate music, gorgeous costumes are loved by many people. In competitive training, sports injuries will reduce the athletic ability of sports dance staff, affect or hinder training plans, and greatly reduce training efficiency. If appropriate and effective treatment measures are not taken, the sports experience of sports dancers will produce a “time bomb.” In sports dance, the negative impact caused by sports injuries has frustrated many players and consumed their original enthusiasm for training. Many sports dancers must give up their original enthusiasm. Sports dance talents choose careers due to injuries and illnesses, which are extremely detrimental to the continuous progress of Chinese sports dance and the sustainable development of the sports dance industry. Therefore, it is necessary to find the cause of the injury and preventive safeguards in time.

The article "Visual Sensor Image Analysis and Massage Techniques to Prevent and Treat Common Injuries of Sports Dance Practitioners" was retracted in 2023. Reasons: signs of a paper mill; suspected computer-generated content; unreliable results or conclusions; concerns about the data.

### 1.2. Related Work

The vision sensor is a specialized vision system with image acquisition and processing and data transmission capabilities. It has become an indispensable key perception method for intelligent industrial robots. Solomon et al. focus on the study of injury treatment and prevention for young dancers. First, it discusses the epidemiology of young dancers' injuries and then describes the screening procedure and sample screening procedures. It then covers physical therapy and resistance training, as well as common diseases and injuries of the spine, hips, knee, and ankle complexes. The conclusion is that preventing young dancers from being injured is important to solve the physical and psychological challenges faced by young performers [1]. Their research is mainly about injury treatment and prevention of young dancers, but the application of visual sensors is insufficient. Geyt et al. mainly evaluate the personal subjective experience of the recipients of cervical spine massage and analyze the influence of kinematics, cavitation, and qualifications of practitioners on personal experience. The method used was to manipulate 20 asymptomatic volunteers on both sides C3 and C5. A 3-dimensional electric goniometer was used to record kinematics, and ISE data was collected through a questionnaire to explore the subject's manipulation experience in touch, relaxation, task perception, and therapist processing. The conclusion is that a better understanding of the individual's subjective experience related to cervical spine massage can increase confidence and improve the doctor-patient relationship and can provide practitioners with further treatment perspectives [2]. Venkatesan and Parthiban proposed that medical image segmentation is a key step in medical image analysis. The methods used are particle swarm optimization (PSO), kernelized FCMPSO (KFCMPSO), optimized fuzzy C-means (FCM), quantum PSO (FCMQPSO), and KFCMQPSO optimized FCM to extract ROI from medical images. The experimental results show that the proposed hybrid FCM and KFCM with PSO and QPSO have good performance and good convergence speed [3]. Moeys et al. introduced the 180-nanometer Towerjazz CIS processing vision sensor named SDAVIS192. By combining the signal-to-noise ratio (SNR) measurements, the characteristics of the DVS event detection threshold are determined, and the results of the black-and-white and RGBW color filter arrays are compared [4]. Luigi mainly studies the prevalence and risk of injuries at the competition and sports level in southeastern France. The method used is to collect data on adolescents (*n* = 1849; 14-19 years old) in French schools in 2015 and 2017. The result obtained is that in almost all sports activities, high-level sports athletes have a higher incidence of injuries than low-level sports athletes [5]. Zhang and Yin pointed out that with high-intensity exercise and training, athletes are increasingly likely to be injured. The common injury parts of sports dancers are waist, knees, shoulders, and ankles. In response to this situation, the authors put forward some suggestions in this article, hoping to effectively alleviate the common sports injuries of aerobics athletes [6]. Although the views put forward by these scholars are accurate, there are still deficiencies in the research process.

The article "Visual Sensor Image Analysis and Massage Techniques to Prevent and Treat Common Injuries of Sports Dance Practitioners" was retracted in 2023. Reasons: signs of a paper mill; suspected computer-generated content; unreliable results or conclusions; concerns about the data.

### 1.3. Innovation

The innovation of this article is as follows: (1) the first is the innovation of the topic selection angle. This article is a new perspective from the perspective of topic selection. At present, there are not many researches that integrate visual sensors, images, massage techniques, sports dance practitioners, common injuries, prevention, and treatment, and it is of exploratory significance. (2) The second is the innovation of research methods. This article puts forward the related technology of a vision sensor image and the related technology of massage, which have high theoretical value and exploratory significance. (3) The other is the innovation of project practice. The results obtained in this article provide a certain reference basis for athletes' injuries, which is convenient for dance practitioners and coaches to better grasp the rules and prevention of injuries in sports dance training and teaching.

## 2. Related Technologies

### 2.1. The Architecture of the Vision Sensor System

The vision sensor system has the following functions. The first is image acquisition and processing, which refers to the acquisition of raw image data through the image sensor and on this basis the use of image registration [7], contour extraction [8], contour fitting, etc. Various image algorithms realize vision application functions such as guided positioning, size measurement [9], barcode recognition [10], and then data interaction, which refers to the remote connection of vision sensors through RS232, TCP/IP, CAN, and other communication methods. Digital image acquisition and processing mainly include three types of depth and color mapping relationships, including true color, false color, and color matching images. Data exchange refers to the integration of several distributed application information systems. Command control, parameter configuration, job file issuance and tool processing results, raw image data, and operating status information of the vision sensor can be transmitted to external devices such as robots, HMI, PLC, and industrial computer through the above-mentioned communication methods. Then, there is graphical programming [11, 12], which refers to the use of graphical programming instead of text programming in the integrated development environment for visual application development. Each visual application tool is an independent module, which can be combined into engineering tasks at will. The file format is issued to the vision sensor. The last is multitask scheduling [13], which means that the vision sensor must perform multiple tasks such as device connection, instruction reception, image acquisition, image processing, and response interruption at the same time, its task priority is different, and it is scheduled based on the priority. To meet the real-time requirements, the overall architecture of the vision sensor system is shown in Figure 1.

The article "Visual Sensor Image Analysis and Massage Techniques to Prevent and Treat Common Injuries of Sports Dance Practitioners" was retracted in 2023. Reasons: signs of a paper mill; suspected computer-generated content; unreliable results or conclusions; concerns about the data.

From top to bottom, the entire system can be divided into a system layer [14], control layer [15], and device layer [16]. Among them, the communication interconnection between the system layer and the control layer is based on various communication interfaces, and the control layer and the device layer are directly connected to the hardware based on the terminal board [17]. The system layer refers to the characteristics of the multilevel state shown by the various elements of the system in the system structure. The control layer is a graphical representation of the relationship between different control levels arranged according to the increasing complexity of the main control system. The equipment floor refers to a certain floor of a high-rise building. All or most of its effective area is used as the layout of equipment such as air conditioning, water supply and drainage, electrical, elevator, and machine room. The hardware architecture of the vision system based on this vision sensor is shown in Figure 2.

### 2.2. Image Fusion Based on Wavelet Transform

Wavelet transform is a new transform analysis method. It inherits and develops the idea of localization of short-time Fourier transform and at the same time overcomes the shortcomings of window size not changing with frequency and can provide a “time-frequency” window that changes with frequency. It is an ideal tool for signal time-frequency analysis and processing. Wavelet transform has the best time-frequency localization characteristics [18], so the method of multiresolution [19] fusion processing of images is becoming increasingly complete with the help of the mathematical tool of wavelet transform [20].

1. Continuous wavelet transform

Let *α*(*x*) be a square integrable function, that is, *α*(*x*) ∈ *W*^2^(*E*); its Fourier transform is $\overset{⌢}{\alpha }\left(g\right)$, if $\overset{⌢}{\alpha }\left(g\right)$ satisfies the following conditions:

(1) $$\begin{array}{c} Q_{\alpha }=\int_{M}{\left|\overset{\wedge }{\alpha }\left(z\right)\right|}^{2}{\left|z\right|}^{-1}sz<\infty , \end{array}$$

Then, *α*(*x*) is called “basic wavelet,” and after *α*(*x*) is stretched and translated, a wavelet sequence can be obtained.

The article "Visual Sensor Image Analysis and Massage Techniques to Prevent and Treat Common Injuries of Sports Dance Practitioners" was retracted in 2023. Reasons: signs of a paper mill; suspected computer-generated content; unreliable results or conclusions; concerns about the data.

For the continuous case, the wavelet sequence is

(2) $$\begin{array}{c} \alpha \left(x\right)=\frac{1}{\sqrt{x}}\alpha \left(\frac{v-b}{a}\right),\;a,b\in R,a\neq 0. \end{array}$$

The expansion factor is a numerical value that characterizes the degree of multicollinearity between the observed values of the independent variables. When the translation factor is within a certain temperature range, the double logarithmic relaxation spectrum measured at any temperature can be superimposed on the relaxation spectrum of the reference temperature by horizontally moving a certain amount of the time logarithmic abscissa. In the formula, *a* is the expansion factor and *b* is the translation factor [21]. In the continuous case, the continuous wavelet transform of any function *u*(*b*) ∈ *Q*^2^(*T*) is defined as

(3) $$\begin{array}{c} K_{z}\left(m,n\right)=<y,\alpha_{m,n}>=\frac{1}{\sqrt{f}}\int_{V}\left(k\right)\dot{\alpha }\left(\frac{v-b}{a}\right)mk. \end{array}$$

Its inverse transformation is

(4) $$\begin{array}{c} u\left(b\right)=\frac{1}{M_{c}}\int_{Q}\int_{Q}\frac{1}{g^{2}}T_{l}\left(m,n\right)\alpha \left(\frac{v-b}{a}\right)vfbh. \end{array}$$

(2) Discrete wavelet transform of the image

The discrete wavelet transform of the image generally uses the two-dimensional Mallat algorithm [22], which can be expressed as

(5) $$\begin{array}{c} e_{m+1}\left(x,y\right)=\underset{l\in T}{\sum }\underset{b\in T}{\sum }k_{1-2n}k_{x-2k}e_{f}\left(l,b\right),\\ D_{k+1}^{1}\left(x,y\right)=\underset{l\in T}{\sum }\underset{b\in T}{\sum }k_{1-2n}m_{b-3n}e_{f}\left(l,b\right),\\ D_{k+1}^{2}\left(x,y\right)=\underset{l\in T}{\sum }\underset{b\in T}{\sum }k_{1+2n}m_{b-3n}e_{f}\left(l,b\right). \end{array}$$

The reconstruction of the image can be expressed as

(6) $$\begin{array}{c} f_{j}\left(x,y\right)\underset{l\in Q}{\sum }\underset{k\in Q}{\sum }{\tilde{h}}_{n-2b}{\tilde{h}}_{v-2c}w_{p+1}\left(l,c\right)+\underset{l\in Q}{\sum }\underset{l\in Q}{\sum }{\tilde{h}}_{n-2b}{\tilde{t}}_{m-2f}{\tilde{R}}_{k+1},\\ g_{k}=\underset{l\in Q}{\sum }\underset{l\in Q}{\sum }{\tilde{k}}_{n-2l}{\tilde{f}}_{m-2b}W_{k+1}^{2}\left(l,b\right)\underset{l\in Q}{\sum }\underset{l\in Q}{\sum }{\tilde{u}}_{b-2l}{\tilde{u}}_{k-2l}T_{p+1}^{3}\left(l,b\right). \end{array}$$

In the formula, $\tilde{k},\tilde{f}$ is a low-pass analysis comprehensive filter and $\tilde{h},\tilde{t}$ is a high-pass analysis comprehensive filter. The synthesis filter uses the same high-quality algorithms as the circuit simulator but is optimized to run quickly and has a gorgeous, fully scalable user interface.

The article "Visual Sensor Image Analysis and Massage Techniques to Prevent and Treat Common Injuries of Sports Dance Practitioners" was retracted in 2023. Reasons: signs of a paper mill; suspected computer-generated content; unreliable results or conclusions; concerns about the data.

### 2.3. Image Fusion Algorithm

1. Evaluation method based on the statistical characteristics of a single image [23]

Suppose the fused image is *Q*(*m*, *n*), the image size is *n* × *n*, and the total gray level is *P*. The average image value reflects the average brightness of the entire image and is also the average gray value of the image, which can be defined as

(7) $$\begin{array}{c} k=\frac{1}{KI}\overset{U-1}{\underset{n=0}{\sum }}\overset{T-1}{\underset{m=0}{\sum }}Q\left(m,n\right). \end{array}$$

In the formula, *Q*(*m*, *n*) is the gray value of the pixel at position (*m*, *n*).

The information entropy of an image is an important indicator to measure the richness of the information contained in the image. The so-called information entropy is a rather abstract concept in mathematics. Here, we might as well understand information entropy as the probability of occurrence of certain specific information, which can represent the value of information. The entropy value [24] reflects the average amount of information contained in the image, which is defined as

(8) $$\begin{array}{c} P=-\overset{K-1}{\underset{o=0}{\sum }}P_{w}\log_{2}e_{z}. \end{array}$$

The information entropy indicates the amount of information contained in the image, and the larger the information entropy, the richer the information of the source image extracted from the fusion image [25].

The standard deviation reflects the discreteness of the image gray relative to the average gray, which is defined as

(9) $$\begin{array}{c} \delta =\sqrt{\frac{\sum_{x=0}^{W-1}\sum_{y=0}^{U-1}{\left[R\left(x,y\right)-r\right]}^{2}}{Z\times E}}. \end{array}$$

The average gradient reflects the sharpness of the image, which is defined as

(10) $$\begin{array}{c} \bar{W}=\frac{1}{Z\times E}\overset{Q}{\underset{b=1}{\sum }}\overset{T}{\underset{v=1}{\sum }}\sqrt{\left[\left(\frac{IR{\left(c,u\right)}^{2}}{Ic}+\left(\frac{IR{\left(c,u\right)}^{2}}{Ib}\right)\right)\right]}. \end{array}$$

The spatial frequency is used to measure the overall activity of the image [26], which is defined as

(11) $$\begin{array}{c} \text{PO}=\sqrt{\frac{1}{\left(U-1\right)\left(R-1\right)}}\overset{X-1}{\underset{x=1}{\sum }}\overset{Y-1}{\underset{y=1}{\sum }}{\left(W\left(x,y+1\right)-W\left(x,y\right)\right)}^{2},\\ \text{ER}=\sqrt{\frac{1}{\left(U-1\right)\left(R-1\right)}\overset{X-1}{\underset{x=1}{\sum }}\overset{Y-1}{\underset{y=1}{\sum }}{\left(W\left(x,y+1\right)-W\left(x,y\right)\right)}^{2},}\\ \text{WT}=\sqrt{{\text{PO}}^{2}+\text{E}{\text{R}}^{2}}. \end{array}$$

(2) Evaluation method based on error sensitivity

Suppose the fusion image and the standard reference image are *W* and *Y*, respectively, and the corresponding images are *W*(*m*, *n*) and *Y*(*m*, *n*), respectively. The root mean square error is defined as [27, 28]

(12) $$\begin{array}{c} \text{RMSE}=\sqrt{\frac{\sum_{x=0}^{X-1}\sum_{y=0}^{Y-1}{\left[W\left(x,y\right)-Y\left(x,y\right)\right]}^{2}}{X\times Y}}. \end{array}$$

The degree of spectral distortion reflects the degree of spectral distortion of the image after fusion, and the expression is

(13) $$\begin{array}{c} {\text{EE}}_{W,Y}=\frac{1}{X\times Y}\overset{X}{\underset{x=1}{\sum }}\overset{Y}{\underset{y=1}{\sum }}\left|W\left(x,y\right)-Y\left(x,y\right)\right|. \end{array}$$

The relative average spectral error (RASE) indicates that the fusion image retains the spectral information of the source multispectral image as follows:

(14) $$\begin{array}{c} \text{RASE}=\frac{1}{X}\sqrt{\frac{1}{Y}\overset{Y}{\underset{k=1}{\sum }}{\text{RMSE}}^{2}\left(T_{e}\right)}. \end{array}$$

The data form of image fusion is an image that contains brightness, color, temperature, distance, and other characteristics of the scene. The correlation coefficient (CC) represents the similarity between the fused image and the source image and is defined as

(15) $$\begin{array}{c} \text{CC}=\frac{\sum_{x=1}^{X}\sum_{y=1}^{Y}\left(W\left(x,y\right)-\partial_{Q}\right)\left(N\left(x,y\right)-\delta_{f}\right)}{\sqrt{\sum_{x=1}^{X}\sum_{y=1}^{Y}{\left(W\left(x,y\right)-\partial_{Q}\right)}^{2}{\left(N\left(x,y\right)-\delta_{f}\right)}^{2}}}. \end{array}$$

The article "Visual Sensor Image Analysis and Massage Techniques to Prevent and Treat Common Injuries of Sports Dance Practitioners" was retracted in 2023. Reasons: signs of a paper mill; suspected computer-generated content; unreliable results or conclusions; concerns about the data.

## 3. Prevention and Research of Sports Dance Injuries

### 3.1. Statistics of Survey Objects and Injury Parts

This article selects 150 injured sports dancers for investigation, including 75 boys and 75 girls. The age of the male player is 22.37 ± 3.12 years, the height is 180.23 ± 3.25 cm, the weight is 67.14 ± 6.21 kg, and the BMI is 21.25 ± 1.51; the age of the female player is 21.25 ± 2.36 years, the height is 167.25 ± 3.56 cm, the weight is 50.2 ± 3.2 kg, and the BMI is 18.21 ± 0.78. According to China's standard female athletes with swords, the BMI is slightly lower than the normal value. This change may be related to the physical requirements of sports dance. However, the BMI value of female athletes is slightly lower than the normal value. Whether it is harmful to the health of female athletes needs further investigation. The statistics of the injured parts of the survey subjects are shown in Table 1.

It can be seen from Table 1 that a survey of 150 sports dancers showed that the waist and knee were injured the most, with an injury rate of 30%, respectively; then, the number of shoulder injuries was the most, with an injury rate of 17%. Then, there were more people with neck injuries, with an injury rate of 13%, followed by toes, with an injury rate of 9%; followed by ankles, with an injury rate of 7%; followed by back, hip, and calf injuries, with an injury rate of 6%; followed by the head and upper limbs, with an injury rate of 5%, respectively; and finally followed by the hip, with an injury rate of 3%. The injury rate of each part of the sports dance athlete's body is shown in Figure 3.

Regardless of the event, for athletes, the waist is the core area of force and the most injured area. In addition, there are many descending and squatting movements in dance. The knee is an important weight-bearing joint of the lower limbs. With a large amount of body weight in the standard dance, the partial load on the knee joint is even greater with the large amount of descent and squatting in the standard dance, and some athletes cannot master the knee joint flow well during training or before the competition. Insufficient knee preparation activities can greatly increase the injury rate of the knee. Statistics of the course of sports injuries in various parts of the body are shown in Table 2.

It can be seen from Table 2 that chronic injuries in the five parts of the body, back, waist, hip, knee, and calf, are clearly more than acute injuries, and some very standardized and delicate dance movements are required in sports dance, and the injured parts are inseparable, so the local load of these parts in dance is relatively large, it is easy to fatigue, and it is easy to cause chronic injuries. The statistics of sports injuries in various parts of the body are shown in Table 3.

It can be seen from Table 3 that most athletes did not completely stop training after being injured.

### 3.2. Gender Differences in Prevalence and Incidence

The popularity rate of Latin dance is higher than that of modern dance, which is closely related to the style of dance. The style of Latin dance is warm and uncontrollable, bold, and rough. Dancers sometimes change the direction and angle radially within a fixed range and sometimes dance together like piano strings. The rhythm is cheerful and energetic, and the hips, upper and lower limbs, and other parts of the body will also move quickly, causing the audience to be overwhelmed. The modern dance style is solemn and elegant and lovely and luxurious, and the dance steps are more standardized and rigorous. Dance partners maintain physical contact to complete various movements and have higher requirements for the knees and ankles. Therefore, the different high exercise intensity, fast movement frequency, and great style characteristics make Latin dance more likely to cause injuries than modern dance, as shown in Table 4 and Figure 4.

The article "Visual Sensor Image Analysis and Massage Techniques to Prevent and Treat Common Injuries of Sports Dance Practitioners" was retracted in 2023. Reasons: signs of a paper mill; suspected computer-generated content; unreliable results or conclusions; concerns about the data.

The prevalence and incidence of different genders are different. Latin dance has the highest prevalence and incidence, followed by ten items. The popularity of Latin dance is higher than that of modern dance. Because the ladies of Latin dance wear high heels and do all kinds of high-intensity and difficult movements, the hip swing and rotating music have a fast rhythm, which affects endurance, speed, and flexibility. In addition, because girls are inherently weaker than boys in terms of natural physiology, it is not difficult to explain that the incidence of female Latin is higher than other items, as shown in Figure 5.

Men and women interpret the characteristics of different styles of dance through different body postures and technical movements in the dance process, and sports injuries often occur in sports. During the past year, there was no significant difference in the nature of the injury ratio between men and women. Muscle strain and ligament strain were the majority, as shown in Table 5.

### 3.3. Prevention and Treatment of Injuries by Manipulation

Tuina is very effective for the injuries caused by sports dance, and Tuina treatment is a very economical method. Let us take the knee joint as an example to discuss the treatment of the knee. Tuina steps are as follows:

In the first step, the patient adopts a straight posture, the doctor stands on the affected side from top to bottom and applies the method to the thigh muscles, inner leg, and back side. Relieve cramps and tension to relieve symptoms completely, and repeat three times for six minutes.

In the second step, the patient takes the supine position and the doctor stands on the affected side. This method relieves the spasm and tension around the thighs and knees to achieve complete relaxation and adjustment and uses traditional massage techniques such as holding and massaging Zen fingers to treat the knee joint, blood Sea, Liangqiu, Knee Inner and Outer Eye, Heding, Yanglingquan, Ashi Point, etc., far acupuncture points, Futu, Zusanli, the penetrating power is strong, and the duration is long. Repeat three times for six minutes.

The article "Visual Sensor Image Analysis and Massage Techniques to Prevent and Treat Common Injuries of Sports Dance Practitioners" was retracted in 2023. Reasons: signs of a paper mill; suspected computer-generated content; unreliable results or conclusions; concerns about the data.

In the third step, the patient takes the supine position. The doctor uses the thumb and hands to act on the affected knee at the same time, pushes the kneecap inward, and fixes it at the same time. Use the compression method to apply a vertical force around the kneecap, and then, use the bottom of the palm to press and rub. Apply even force to the lower end of the kneecap. Inhale and endure, with the accumulation of acid as the gas level, and repeat three times for approximately six minutes.

In the fourth step, the doctor moves the affected knee joint and instructs the patient to actively bend, extend, rotate, and abduct. Finally, we use diathermy to rub around the knee joint for six minutes. Once a day, seven times a course of treatment, one day between the two courses of treatment, a total of four weeks of treatment, the anatomical parts selected by the observation point of the body surface temperature outside the knee joint and the posterior anterior side are shown in Figure 6.

When selecting observation points for body surface temperature changes, to facilitate statistical data and intuitive comparison of specific data on body surface temperature changes between the two groups, select the infrared temperature observation images of body surface temperature before and after noon treatment in the massage group and the traditional massage group: comprehensive observation. Record and compare the obvious anatomical position of the monitoring section around the knee joint, and use its specific anatomical position as the unique name of the temperature monitoring point. The determination of the sedimentation observation period should be based on the principle that it can systematically reflect the change process of the measured sedimentation without omitting its change time, and it should be determined according to the amount of sedimentation per unit time and the degree of external influence.

## 4. Experimental Results and Analysis

### 4.1. WOMAC Score

After the WOMAC score and statistical analysis of the two groups of patients, the results: the pain, and stiffness of the patients before treatment, the total score of daily activity disorder was compared with each other (*P* > 0.1), which was not statistically significant. After treatment, the total scores of pain, stiffness, and disturbance of daily activities of the patients were compared with each other (*P* > 0.1), which was not statistically significant. Before treatment, the total scores of pain, stiffness, and dysactivity of the two groups of patients were compared before and after the treatment (*P* < 1); there was a significant statistical difference, indicating that the two treatment methods have achieved significant effects, and the scores are shown in Figure 7.

The article "Visual Sensor Image Analysis and Massage Techniques to Prevent and Treat Common Injuries of Sports Dance Practitioners" was retracted in 2023. Reasons: signs of a paper mill; suspected computer-generated content; unreliable results or conclusions; concerns about the data.

Compared with the traditional two groups of patients, the body surface observation point temperature after treatment is better than that of the traditional group (*P* < 0.1); there is a difference between these two groups. Compared with the body surface observation point temperature before and after treatment, the difference between the Jingjin group and the traditional group was statistically significant. Comparing the changes in body surface temperature at the observation point, it can be determined that the temperature of the preoperative body surface temperature observation point in the Jingjin group and the traditional massage group is very different from that after the treatment. After the treatment, it has no obvious effect on the comparison. The knee of patients with knee osteoarthritis is subjected to infrared thermal imaging. The thermal image is shown in Figure 8.

In the meridian massage group, 18 cases were cured, 46 cases were markedly effective, 8 cases were improved, and 3 cases were not healed. The total effective rate was 96%; in the traditional massage group, 15 cases were cured, 41 cases were markedly effective, 13 cases were improved, and 6 cases were not healed. The efficiency is 92%. The chi-square test showed a statistical difference (*P* < 0.1), and the curative effect of the meridian massage group was significantly better than that of the traditional massage group.

### 4.2. Analysis of the Main Causes of Sports Injuries

1. Poor physical fitness

According to statistics, in the questionnaire survey of coaches and athletes, sports injuries caused by poor physical condition are the primary factor among all injury factors. This shows that both Chinese dance coaches and athletes believe that poor physical condition is the most important factor leading to sports injuries. Among them, strength accounts for more than half of the injury rate, followed by flexibility, endurance, and coordination. Judging from this ratio, it seems that Chinese dancers do not pay enough attention to the training of strength and flexibility.

(2) Incorrect technical essentials and deviation of foot focus

If the toe opening is too large, it will cause the midsection of the hip to leak out to the side, and it will not be able to better support forward movement. When the athlete performing the Latin dance is standing and walking, everyone has different opinions regarding the angle of the toe. When dancing, most people usually focus on the inside of the big toe. The human foot is composed of multiple bones and soft tissues, supporting the weight of the erect person. The data of the toe opening angle and the main focus points of the foot are shown in Figure 9.

(3) Improper coordination and cooperation between dance partners

The male partner's choice of dance steps, changes in movement orientation, and performance of dance styles must be mastered and can be used actively, quickly, decisively, and accurately. Female partners are required to have an agile following ability to accurately accept the dance signals given by the male partner, to quickly and accurately change their dance steps and postures, and to go with the flow, cooperate very actively and easily, complete each dance step, and dance. In the process, the female partner should not overpower the guests or change the dance steps at will or she should not subjectively speculate or guess the movement of the dance steps; otherwise, it is prone to mutual collision and disconnection of the lead band and unnecessary sports injuries.

(4) Unreasonable warm-up activities

Heating is to improve the stimulation of the central nervous system through low-intensity to moderate-intensity exercise to reach an appropriate level, strengthen the activities of different organs, overcome various functional inactivities, improve the temperature and functional flexibility of muscles and tissues, strengthen dependent reflex contact, promote rapid recovery of the human body, and prepare for formal training. At the same time, it is also one of the important measures to prevent sports injuries.

(5) Failure to receive timely treatment and positive adjustment for injury training

Dancers do not know how to reflect their physical condition, or under the strict requirements of coaches, they dare not truthfully report their physical condition, but stick to it. High-load and intense practice is easy to make coaches and athletes difficult to detect the warning signals sent by the body. Therefore, in training, when the players are injured and the symptoms are not very obvious, they often do not receive medical treatment in time.

(6) External factors causing damage

According to further investigations, the main reasons for sports dancers' injuries are as follows: characteristics of Latin dance events, excessive local weight-bearing, neglect of recovery after exercise, excessive exercise load, insufficient preparation activities, improper training methods, failure to pull after training stretching, unreasonable use of technology, poor physical condition, and inappropriate dance shoes or dance clothes, as shown in Figure 10.

The article "Visual Sensor Image Analysis and Massage Techniques to Prevent and Treat Common Injuries of Sports Dance Practitioners" was retracted in 2023. Reasons: signs of a paper mill; suspected computer-generated content; unreliable results or conclusions; concerns about the data.

## 5. Conclusions

Through the research in this article, it is found that the number of people with waist and knee injuries is the largest, with an injury rate of 30%, followed by the number with shoulder injuries, with an injury rate of 17%; followed by more people with neck injuries, with an injury rate of 13%; followed by the toes, with an injury rate of 9%; followed by the ankle, with an injury rate of 7%; followed by the back, hip, and calf injuries, with an injury rate of 6%; and followed by the head, face, and upper limbs, with an injury rate of 5%, respectively. Finally, the hip has an injury rate of 3%. The reason for the injury is that there is no warm-up session before the exercise or the warm-up session is perfunctory; the athlete's technical level is poor; the physical fitness is poor; the training method is unscientific; the amount of exercise and exercise intensity are too large; the training schedule is unreasonable and the time is too long; athletes choose difficult dance moves that do not meet their own level; there is no coordination between male and female athletes; athletes select unreasonable music rhythm; there is physical decline during the competition; they are unable to adjust their own state reasonably before the competition; and collisions with other players happen during the competition. They are all causes of sports injuries of sports dancers in Xi'an. In response to this, our proposed massage technique has certain advantages over western medicine's oral medicine in terms of cure rate and improvement rate, and it avoids the burden and harm to the patient's body and economy caused by surgical treatment and joint cavity injection. In the future, we need to continue to sum up the experience, ingeniously combine modern technology and equipment, and explore increasingly effective comprehensive therapies on the basis of research on the treatment mechanism of Chinese medicine, to improve the cure rate, relieve the suffering of patients, and use traditional Chinese medicine such as massage and acupuncture. We think that in the future, Tuina technology will have a very critical impact on many medical diseases. Tuina technology will also collide with more technologies to produce new treatment technologies.

## Figures and Tables

**Figure 1:** Vision sensor system architecture.

**Figure 2:** Vision system hardware architecture based on vision sensors.

**Figure 3:** Injury rate of sports dancers in various parts of the body.

**Figure 4:** Statistics of prevalence and incidence of different dance styles.

**Figure 5:** Statistics on the prevalence and incidence of male and female dances of different genders.

**Figure 6:** The selected anatomical parts of the body surface temperature observation point outside the posterior anterior side of the knee joint.

**Figure 7:** WOMAC scores of the two groups of patients before and after treatment.

The article "Visual Sensor Image Analysis and Massage Techniques to Prevent and Treat Common Injuries of Sports Dance Practitioners" was retracted in 2023. Reasons: signs of a paper mill; suspected computer-generated content; unreliable results or conclusions; concerns about the data.

**Figure 8:** Infrared thermal imaging of the knee of a patient with knee osteoarthritis.

**Figure 9:** The angle of the toe opening and the main focus of the foot.

**Figure 10:** Causes of sports injuries.

**Table 1:** Injury statistics of various parts of the body of sports dancers.

Injury site	Number of injured
Head face	8
Neck	20
Shoulder	25
Upper limb	8
Back	10
Waist	45
Buttocks	10
Hip	5
Lap	45
Calf	10
Ankle	11
Toes	14

**Table 2:** Statistics of the course of sports injuries in various parts of the body.

Injury site	Acute injury	Chronic injury
Head face	5	4
Neck	8	12
Shoulder	9	15
Upper limb	3	2
Back	2	9
Waist	8	36
Buttocks	2	10
Hip	2	5
Lap	14	30
Calf	4	12
Ankle	14	12
Toes	13	10

**Table 3:** Statistics on the degree of sports injury in various parts of the body of sports dancers.

Injury site	Number of injured	Number of people who stopped training completely	%	Partially stopped training	%	Normal training number	%
Head face	8	1	12.2%	2	13.2%	6	72.6%
Neck	20	1	0	6	25%	15	75%
Shoulder	25	0	0	4	14%	19	45%
Upper limb	8	0	4.5%	3	45%	3	40%
Back	10	0	18%	3	20%	8	71.5%
Waist	45	1	8.5%	7	12%	32	72.6%
Buttocks	10	1	9%	2	14%	8	45%
Hip	5	2	10%	2	12.5%	2	52%
Lap	45	4	0	8	15%	32	64.3%
Calf	10	0	8.5%	6	14.3%	10	48.6%
Ankle	11	1	7%	12	25.6%	14	66.5%
Toes	14	1	0	8	40.2%	19	48.6%
Injury site	8	2	11%	12			

**Table 4:** Statistics of the number of injured parts.

	Neck	Shoulder and elbow	Chest and abdomen	Waist	Back	Buttocks	Hip bone	Lap	Neck
Latin	1	2	0	3	2	0	0	1	4
Modern	2	0	0	1	3	0	0	2	0
Total	3	2	0	4	5	0	0	3	4

**Table 5:** The nature and number of sports and dance injuries of male and female players.

Nature of injury	Boys	Girls	Total
Muscle strain	4	8	12
Ligament strain	3	5	8
Osteochondrosis	0	2	2
Herniated disc	0	2	2
Joint dislocation	0	0	0
Meniscus injury	0	0	0
Fracture	1	0	1
Periostitis	3	3	6
Tendon sheath	2	2	4
Antibursitis	0	0	0
Total	13	22	35

## Data Availability

Data sharing is not applicable to this article as no datasets were generated or analyzed during the current study.
